The article "Comparison of the Efficacy of the Panoramic and Cone Beam Computed Tomography Imaging Methods in the Surgical Planning of the Maxillary All-On-4, M-4, and V-4" was published in 2022. Journal: Biomed Res Int.

# Comparison of the Efficacy of the Panoramic and Cone Beam Computed Tomography Imaging Methods in the Surgical Planning of the Maxillary All-On-4, M-4, and V-4

**DOI:** 10.1155/2022/1553340

**Published:** 2022-07-27

**Authors:** Erim Tandogdu, Aysa Ayali, Mehmet Gagari Caymaz

**Affiliations:** ^1^Department of Oral and Maxillofacial Surgery, Near East University Faculty of Dentistry, Nicosia, Mersin 10, Turkey; ^2^Department of Oral and Maxillofacial Surgery, European University of Lefke Faculty of Dentistry, Lefke, Mersin 10, Turkey; ^3^Department of Oral and Maxillofacial Surgery, Cyprus Health and Social Sciences University Faculty of Dentistry, Morphou, Mersin 10, Turkey

## Abstract

This study is aimed at analyzing the difference between the measurements made according to certain anatomical signs of the maxillary jaw using panoramic radiography and cone beam computed tomography (CBCT) to decide whether to use all-on-4, M-4, or V-4 configuration to prevent complications caused by incorrect measurements during the presurgical planning stage of the placement of implants in the all-on-4 technique. A retrospective study was conducted with 50 patients with upper edentulous jaws suitable for the all-on-4 technique, who underwent preoperative panoramic radiography and cone beam computed tomography evaluation for dental implant surgery. The shortest vertical distances between anatomical structures were measured. Measurements were made independently by two oral and maxillofacial surgeons, one experienced and the other inexperienced. A statistically significant difference was found between the mean values according to gender (*p*=0.045). When the measurements made by the experienced surgeon and the inexperienced surgeon were compared, there was no significant difference between panoramic radiography and cone beam computed tomography. In situations where bone measurements are required for deciding on all-on-4 or one of its configurations (M-4 and V-4), it was found that panoramic radiography gives significantly incorrect results compared to cone beam computed tomography (*p*<0.05). Cone beam computed tomography is more reliable than panoramic radiography and eliminates the margin of error in the planning of all-on-4 or its variations to be made by either an experienced or an inexperienced oral surgeon.

## 1. Introduction

Dental implants are regarded as the main treatment option in terms of rehabilitation of edentulous jaws because of their stable results and satisfactory success rates [1, 2]. In the all-on-4 treatment concept, a total of four implants are to be placed to withstand a full-arch prosthesis [3]. The implants, both anterior and posterior, converge towards the apex in angulation of 30 degrees. The apical divergence of the implants allows an increase in the anteroposterior spread, leading to improved prosthetic load distribution [4]. From a biomechanical viewpoint, at least 10 mm of bone height is needed in the anterior maxilla to allow the fixed implant-supported prosthesis to be immediately loaded [3]. Nevertheless, this is not always achievable because augmentation of bone height is a complex challenging surgical procedure, especially in the anterior maxilla areas with severe atrophy. In patients whose smile-line is high, the maxillary alveolar bone should be reduced to move the horizontal transition line apically to achieve an esthetically satisfactory result [4]. Such clinical situations could lead to inadequate alveolar bone height in the anterior maxilla, consequently obstructing the axial placement of at least 10 mm implants. As a result, inclining the anterior implants permits longer implants to be placed distally, following the guidelines of the all-on-4 concept. Jensen and Adams [3] introduced an M-shaped design, called the M-4, where the anterior implants are tilted up to 30 degrees distally in the axial plane while extending into the lateral nasal rim. The other design, called the V-4, is composed of four implants that are tilted in the direction of the midline in a V-shaped figure, where the anterior two implants engage apically in the maxillary midplane [4].

The article "Comparison of the Efficacy of the Panoramic and Cone Beam Computed Tomography Imaging Methods in the Surgical Planning of the Maxillary All-On-4, M-4, and V-4" was published in 2022. Journal: Biomed Res Int.

In treatment planning, the constantly used imaging methods are panoramic radiography, intraoral radiography, computed tomography (CT), and cone beam computed tomography (CBCT) [5]. From these modalities, panoramic radiography is usually used due to its advantages of providing cost-efficient, easily obtainable, and high-quality images [6]. CBCT not only acquires large amounts of data on relatively short exposure to radiation but also yields high-resolution images in multiple orthogonal planes, which is helpful for accurate measurements [7].

Even though a substantial number of publications are available on the applications of CBCT and panoramic radiography in dental implantology, there is still debate regarding the ideal imaging method for presurgical implant planning [8].

Therefore, the present study is aimed at analyzing the difference between the measurements made according to certain anatomical signs of the maxillary jaw using panoramic radiography and CBCT to decide whether to use all-on-4, M-4, or V-4 configuration to prevent complications caused by incorrect measurements during the presurgical planning stage of the placement of implants in the all-on-4 technique. It is also aimed at comparing the measurements of a senior (experienced) and a junior (inexperienced) oral surgeon to evaluate whether experience significantly affects making an accurate measurement.

The article "Comparison of the Efficacy of the Panoramic and Cone Beam Computed Tomography Imaging Methods in the Surgical Planning of the Maxillary All-On-4, M-4, and V-4" was published in 2022. Journal: Biomed Res Int.

The first hypothesis in the current study is that there will be a notable difference between the CBCT and panoramic radiography measurements, and the second null hypothesis is that there will be a difference between the measurements of an experienced and an inexperienced oral surgeon in these measurements.

## 2. Materials and Methods

### 2.1. Ethical Considerations

The study protocol was approved by the Near East University Scientific Research Ethics Committee (project number NEU/2019/89-1304).

### 2.2. Study Setting and Grouping of Participants

A retrospective study was conducted in the Near East University Faculty of Dentistry Department of Oral and Maxillofacial Surgery with 50 patients (58% of the patients were male and 42% were female). The mean age of the patients was 62: the minimum age was 22 and the maximum age was 92, with upper edentulous jaws suitable for the all-on-4 technique, who had preoperative panoramic radiography and CBCT assessment for dental implant surgery between September 2016 and August 2021.

Subsumption criteria were panoramic radiography and CBCT images showing the maxillary edentulous region clearly. Images showing artifacts, geometric distortion, and indeterminate anatomical structures were excluded from the study data [9].

CBCT images were captured using Sirona Orthophos SL® 3D (Sirona, Salzburg, Austria) with 85 kV voltage, 6 mA current, 16 × 5 cm scan area, and 14 sec. Scan time also panoramic radiographs were taken using the Orthophos XG® (Sirona, Salzburg, Austria) using 1.2 magnification, 60 kV voltage, 4 mA current, and exposure time of 14 sec. All measurements were performed using the same software program Sirona Sidexis® v.4 (Sirona, Salzburg, Austria).

Panoramic images at 1 : 1 magnification and on CBCT scans were viewed in the coronal and sagittal planes. The vertical distances between anatomical structures were measured as follows:

1. Distance between the right and left nasal floors (Figure 1)
2. Distance between the right/left lateral nasal wall and right/left maxillary sinus (Figure 2)
3. Distance between the bottom of the left and/or right nasal floor and the alveolar crest (Figure 3)
4. Distance between the right/left maxillary lateral incisor tooth region and the right/left maxillary first molar tooth region (Figure 4)
5. Distance between the right and left maxillary lateral incisor tooth region (Figure 5)

The measurements were made, at the Near East University Faculty of Dentistry Department of Oral and Maxillofacial Radiology, independently on the same monitor and under equal examining conditions by two oral and maxillofacial surgeons, one experienced (more than 10 years in the field) and the other inexperienced (less than 5 years in the field). Measurements obtained from each patient were recorded in mm. All examinations and measurements were performed on a 60.5 cm, 1920 × 1080 resolution, 23.8-inch color LCD (liquid crystal display) monitor (Acer ET241Y, Acer Corporation, New Taipei City, Taiwan), under subdued room lighting.

The article "Comparison of the Efficacy of the Panoramic and Cone Beam Computed Tomography Imaging Methods in the Surgical Planning of the Maxillary All-On-4, M-4, and V-4" was published in 2022. Journal: Biomed Res Int.

### 2.3. Statistical Analysis

Data were analyzed with IBM SPSS V23. Relevance to normal distribution was evaluated by the Kolmogorov-Smirnov test. One-way analysis of variance was used in the comparison of normally distributed data according to groups of three or more, and multiple comparisons were performed with the Tukey HSD test. An independent two-sample *t*-test was used to compare normally distributed data according to paired groups. Analysis results were presented as mean ± standard deviation and median (minimum-maximum) for quantitative data. The significance level was taken as *p* < 0.050.

## 3. Results

After evaluating the eligibility criteria, the final sample consisted of 29 men (58%) and 21 women (42%) aged between 22 and 92 (mean 62 years). A statistically significant difference was found between the mean values of the lateral nasal wall and maxillary sinus (right) according to gender (*p* = 0.045). The mean for women was 5.5, while the mean for men was 6.0. A statistically significant difference was found between the mean values of the lateral nasal wall edge—maxillary sinus (left) according to gender (*p* = 0.003). The mean for women was 5.3, while the mean for men was 6.1. A statistically significant difference was found between the mean values of the lateral incisor region (left) and lateral incisor region (right) according to gender (*p* = 0.03). The mean for women was 16.7, while the mean for men was 17.7. A statistically significant difference was found between the mean values of the nasal floor and the alveolar crest (left) by gender (*p* = 0.021). While the average for women was 12.9, the average for men was 14.1. There was no statistically significant difference between the mean values of other variables by gender (*p* > 0.050). The mean values of the distances by gender in panoramic radiography and CBCT images are shown in Table 1.

When the measurements made by the experienced surgeon and the inexperienced surgeon were compared, there was no significant difference between panoramic radiography and CBCT (*p* < 0.001). However, there was a difference between all measurement regions in panoramic radiography and CBCT measurements. The mean values of the measurements are presented in Table 2.

The article "Comparison of the Efficacy of the Panoramic and Cone Beam Computed Tomography Imaging Methods in the Surgical Planning of the Maxillary All-On-4, M-4, and V-4" was published in 2022. Journal: Biomed Res Int.

In situations where bone measurements are required for deciding on all-on-4 or one of its configurations (M-4 and V-4), it was found that panoramic radiography gives significantly incorrect results compared to CBCT (*p* < 0.05) (Table 3).

In the CBCT, according to the experienced surgeon, 12 out of a total of 50 cases were found to have a nasal floor—alveolar crest (left) distance value of <10. So, 24% of all-on-4 cases should be done with M-4 and V-4 configurations. When looking at the anterior-posterior (A–P) distance, 10% of all-on-4 cases were found to be suitable for the M-4 configuration and 14% for the V-4 configuration. In the panoramic radiography group evaluated by the experienced surgeon, only 3 cases were found <10. In other words, 9 cases were incorrectly measured.

In the CBCT group evaluated by the inexperienced surgeon, 11 of a total of 50 cases were found to have a nasal floor—alveolar crest (left) distance value of <10. Accordingly, 22% of all-on-4 cases should be done with the M-4 and V-4 configurations. When looking at the A–P distance, 2% of all-on-4 cases were found to be suitable for the M-4 configuration, and 20% for the V-4 configuration. In the panoramic radiography group evaluated by the inexperienced surgeon only 3 cases were found <10. In other words, 8 cases were incorrectly measured.

No statistically significant difference was found between the distributions of lateral incisor region—first molar region (right) according to the nasal floor—alveolar crest (right) condition in each group (*p* > 0.050) in Table 4.

In the experienced surgeon CBCT group, in 13 out of 50 cases, the nasal floor—alveolar crest (right) distance value was <10. So, 26% of all-on-4 cases should be done with the M-4 and V-4 configurations. When looking at the A–P distance, it was seen that 6% of all-on-4 cases were suitable for the M-4 configuration, and 20% for the V-4 configuration. In the experienced surgeon panoramic group, only 3 cases were found. In other words, 10 cases were incorrectly measured (Table 5).

In the inexperienced surgeon CBCT group, of the total 50 cases, 10 had a nasal floor—alveolar crest (Right) distance value of <10. That is, 20% of all-on-4 cases should be done with the M-4 and V-4 configurations. When looking at the A–P distance, 4% of all-on-4 cases were suitable for the M-4 configuration, and 16% for the V-4 configuration. In the inexperienced surgeon panoramic group, only 3 cases were found. In other words, 7 cases were incorrectly measured (Table 5).

## 4. Discussion

Different imaging techniques are available in maxillofacial radiology. Intraoral radiographs, panoramic radiographs, and CBCT are the most favored techniques in dental implant surgeries.

The article "Comparison of the Efficacy of the Panoramic and Cone Beam Computed Tomography Imaging Methods in the Surgical Planning of the Maxillary All-On-4, M-4, and V-4" was published in 2022. Journal: Biomed Res Int.

The 2-dimensional (2D) nature of intraoral radiographs can cause anatomical proposition and dimensional distortion [10]. Isidor expressed that because of superimposition, it was not feasible to spot an inadequate marginal bone height or lack of osseointegration on 2D images [11]. In addition, many types of research have proven that the limited preoperative diagnostic capability of 2D imaging modality in dental implantology can cause implant failure [12]. 2D images demonstrate interproximal alveolar bone levels in the orovestibular direction, which is a key specification for following the peri-implant bone [13].

Panoramic radiographs enable a detailed 2D inspection of the jaws. The most important benefits of panoramic radiographs are a low radiation dose, comparatively lesser time of exposure, and clarity of examination [14]. On the other hand, the lower image quality in comparison to intraoral radiographs and the existence of ghost images are some of the disadvantages of panoramic radiography [15]. Laster et al. published that in panoramic radiography as a result of distortion and overlapping, horizontal measurements can be questionable [16].

CBCT, which is another imaging method and provides 3-dimensional (3D) examination has been the choice of use in dental implant surgeries [7]. CBCT is favorable as a result of its high spatial resolution, short scanning time, and rapid image obtaining [17].

The results of implant treatment have become quite expectable in recent years [18]. However, the relationship of implants to fundamental vital anatomy landmarks can considerably alter the success of the surgical operation. Therefore, implant failure could limit the preoperative diagnostic examination to the panoramic imaging method [12]. Tang et al. proposed that in situations where implant surgery presents any risks of damage to vital structures, using 3D imaging techniques could be advantageous [15]. Similarly, Dreiseidler et al. stated that the image quality of CT and CBCT is higher than panoramic radiography, but they are not being acquirable in every hospital because of their technical requirements and high cost are the main disadvantages of these imaging methods [19]. Besides that, Monsour and Dudhia proposed that patients experiencing CT examinations were exposed to a higher radiation dose than those who underwent examinations using panoramic radiography and CBCT [20].

On the other hand, one of the main problems associated with dental implant surgeries is the recovery of patients with extremely atrophic maxilla [21]. Clinical research related to the number of implants required for rehabilitation of the edentulous jaws discovered the use of four implants led to an equivalent success level to rehabilitation processes with more implants [22, 23]. Jensen et al. say that inclining anterior implants may also affect the identical pattern as inclining posterior implants which permits positioning of 50% longer implants [24]. There are two alignments with these features that have been reported. The first form is the M-4 design, in which the anterior implants are tilted posteriorly in the axial plane up to 30 degrees, reaching the lateral nasal rim. The second form, named V-4, which inserted in a V-shaped form and includes four implants that are angled to the midplane, with the two anterior implants apically joined in the maxillary midline [25].

The article "Comparison of the Efficacy of the Panoramic and Cone Beam Computed Tomography Imaging Methods in the Surgical Planning of the Maxillary All-On-4, M-4, and V-4" was published in 2022. Journal: Biomed Res Int.

Jensen and Adams in their research stated that compared to the standard all-on-4 configuration, the M-4 method could have more mechanical benefits and it is the choice for clinicians to achieve implant durability without exposing patients to further surgeries [3]. He suggested that in maxillae when there is sufficient bone mass posterior to the nasal cavity, we should use the M-4 configuration, but when the anteroposterior bone mass is not adequate and is limited to the inter-canine area the V-4 configuration should be used [3, 4].

When primary stability is of concern, all-on-4 different variations with tilted anterior implants can be considered beneficial because of the insertion of longer implants. Therefore, in this study, the standard all-on-4 treatment concept and its variations, which are intended to be applied to patients with severely atrophic maxilla, were compared in terms of applicability with panoramic radiography and CBCT between the inexperienced surgeon and the experienced surgeon. In the CBCT, according to the experienced surgeon, 12 out of a total of 50 cases were found to have a nasal floor—alveolar crest (left) distance value of <10. So, 24% of all-on-4 cases should be done with M-4 and V-4 configurations. When looking at the A–P distance, 10% of all-on-4 cases were found to be suitable for the M-4 configuration and 14% for the V-4 configuration. In the panoramic radiography group evaluated by the experienced surgeon, only 3 cases were found <10. In other words, 9 cases were incorrectly measured. In the experienced CBCT group, in 13 out of 50 cases, the nasal floor—alveolar crest (right) distance value was <10. So, 26% of all-on-4 cases should be done with the M-4 and V-4 configurations. When looking at the A–P distance, it was seen that 6% of all-on-4 cases were suitable for the M-4 configuration, and 20% for the V-4 configuration. In the experienced surgeon panoramic group, only 3 cases were found. In other words, 10 cases were incorrectly measured. In the CBCT group evaluated by the inexperienced surgeon, 11 of a total of 50 cases were found to have a nasal floor—alveolar crest (left) distance value of <10. Accordingly, 22% of all-on-4 cases should be done with the M-4 and V-4 configurations. When looking at the A–P distance, 2% of all-on-4 cases were found to be suitable for the M-4 configuration, and 20% for the V-4 configuration. In the panoramic radiography group evaluated by the inexperienced surgeon only 3 cases were found <10. In other words, 8 cases were incorrectly measured. In the inexperienced surgeon CBCT group, of the total 50 cases, 10 had a nasal floor—alveolar crest (right) distance value of <10. That is, 20% of all-on-4 cases should be done with the M-4 and V-4 configurations. When looking at the A–P distance, 4% of all-on-4 cases were suitable for the M-4 configuration, and 16% for the V-4 configuration. In the inexperienced surgeon panoramic group, only 3 cases were found. In other words, 7 cases were incorrectly measured.

The article "Comparison of the Efficacy of the Panoramic and Cone Beam Computed Tomography Imaging Methods in the Surgical Planning of the Maxillary All-On-4, M-4, and V-4" was published in 2022. Journal: Biomed Res Int.

This shows that in the majority of cases, it was determined that it was more suitable for the V-4 concept due to the short A–P distance. At the same time, it was seen that the measurements made by the inexperienced surgeon and the experienced surgeon on panoramic radiography were similar and the margin of error was higher than that of CBCT. That is, CBCT has a lower margin of error to measure the A–P distance while planning all-on-4.

In different research that supports our study, Tang et al. compared the magnification rate of CBCT and panoramic radiography in the assessment of various maxillofacial loci and stated that the distances calculated by panoramic radiography were closely correlated with those assessed by CBCT [15]. In such cases, using CBCT is recommended for more precise planning even though this study reveals that the average difference between CBCT and panoramic radiography was less than 1 mm.

Using of various imaging modalities for preimplant assessment has been analyzed in numerous researches. Kopecka et al. compared the use of CBCT and panoramic radiography in the evaluation of the bone height present for dental implant insertion surgeries [26]. In post-mortem research, Hu et al. used the maxillary region to compare measurement errors on CBCT images and panoramic radiographs and discovered that the average presurgical measurement error was significantly higher for panoramic radiography than CBCT [27]. In his research, no statistically significant difference was found between the measurements made by the inexperienced oral surgeon and the experienced oral surgeon on panoramic radiography. However, a statistically remarkable difference was found between the values in CBCT measurements.

The article "Comparison of the Efficacy of the Panoramic and Cone Beam Computed Tomography Imaging Methods in the Surgical Planning of the Maxillary All-On-4, M-4, and V-4" was published in 2022. Journal: Biomed Res Int.

This study's primary limitation was the number of the cases selected for the study. This limitation was due to the limited number of maxillary edentulous population in our university and we tried to present all scans using the same software. The cases were selected between September 2016 and August 2021. In addition, each measurement has been done once, and by making more measurements, we can obtain a detailed average for each region.

## 5. Conclusions

Within the study's limitations, we can conclude that CBCT is more reliable than panoramic radiography and eliminates the margin of error in the planning of all-on-4 or its variations (M-4 and V-4) to be made by either an experienced or an inexperienced oral surgeon. Further studies should review the availability of computer-aided implant surgery with a surgical guideline based on CBCT.

## Figures and Tables

**Figure 1:** Measurement of the shortest vertical distance between the right and left nasal floors on a panoramic image (a) and a cone beam computed tomography image (b).

**Figure 2:** Measurement of the shortest vertical distance between the left lateral nasal wall and left maxillary sinus on a panoramic image (a) and a cone beam computed tomography image (b).

**Figure 3:** Measurement of the shortest vertical distance between the bottom of the nasal floor and the alveolar crest on a panoramic image (a) and a cone beam computed tomography image (b).

**Figure 4:** Measurement of the shortest vertical distance between the maxillary lateral incisor tooth region and the maxillary first molar tooth region on a panoramic image (a) and a cone beam computed tomography image (b).

**Figure 5:** Measurement of the shortest vertical distance between the right and left maxillary lateral incisor tooth region on a panoramic image (a) and a cone beam computed tomography image (b).

**Table 1:** Comparison results by gender.

	Gender		Total	Test statistics	*p*
	Female	Male			
Between nasal floors	11,9 ± 2,3	12,4 ± 2,3	12,2 ± 2,3	*t* = −1,728	0.085
	12,1(4,1-16,1)	12,3 (5,8-18,0)	12,3 (4,1-18,0)		
Nose edge—maxillary sinus (right)	5,5 ± 1,7	6,0 ± 2,1	5,8 ± 2,0	*t* = −2,021	0.045
	5,4 (1,8-9,0)	5,8 (2,7-11,8)	5,5 (1,8-11,8)		
Nose edge—maxillary sinus (left)	5,3 ± 1,6	6,1 ± 1,8	5,8 ± 1,7	*t* = −3,051	0.003
	5,2 (2,3-9,4)	6,0 (2,3–11,0)	5,5 (2,3-11,0)		
Lateral incisor region—first molar region (left)	19,1 ± 3,6	20,1 ± 4,3	19,7 ± 4,1	*t* = −1,697	0.091
	18,2(11,2-271)	20,2 (8,3-28,0)	19,5 (8,3-28,0)		
Lateral incisor region—first molar region (right)	19,0 ± 3,3	19,7 ± 4,3	19,4 ± 3,9	*t* = −1,296	0.196
	19,1(9,6-27,5)	19,7 (5,3-28,9)	19,4 (5,3-28,9)		
Lateral incisor region (left)—lateral incisor region (right)	16,7 ± 2,9	17,7 ± 3,1	17,3 ± 3,0	*t* = −2,182	0.030
	16,9(8,9-22,9)	17,7(11,1-26,1)	17,5 (8,9-26,1)		
Nasal floor—alveolar crest (right)	12,9 ± 3,8	13,8 ± 3,4	13,4 ± 3,6	*t* = −1,723	0.086
	12,8(5,1-21,2)	13,8 (5,8-24,7)	13,3 (5,1-24,7)		
Nasal floor—alveolar crest (left)	12,9 ± 3,8	14,1 ± 3,6	13,6 ± 3,7	*t* = −2,334	0.021
	12,8(5,3-22,0)	13,7 (5,4-25,4)	13,3 (5,3-25,4)		

Note: *t*: independent *t*-test for two samples. Data are presented as *mean* *value* ± *standard* *deviation*/median (minimum-maximum) in millimeter.∗*p* < 0.05 indicates a significant difference.

The article "Comparison of the Efficacy of the Panoramic and Cone Beam Computed Tomography Imaging Methods in the Surgical Planning of the Maxillary All-On-4, M-4, and V-4" was published in 2022. Journal: Biomed Res Int.

**Table 2:** Comparison results by groups.

	Group				Test statistics	*p*
	Experienced Panoramic	Experienced CBCT	Inexperienced Panoramic	Inexperienced CBCT		
Between nasal floors	13,4 ± 2,0b	11,5 ± 1,7a	13,4 ± 2,0b	10,5 ± 2,2a	*F* = 25,711	<0.001
	13,5	11,3	13,5	10,5		
	(9,8-18,0)	(8,5-15,3)	(9,8-17,9)	(4,1-14,1)		
Nose edge—maxillary sinus (right)	6,5 ± 2,0b	5,4 ± 1,8a	6,6 ± 1,7b	4,9 ± 1,5a	*F* = 9,138	<0.001
	6,4	5,3	6,4	4,8		
	(2,4-11,2)	(1,8-11,8)	(2,4-11,2)	(2,3-11,8)		
Nose edge—maxillary sinus (left)	6,5 ± 1,7b	5,2 ± 1,5a	6,5 ± 1,7b	4,9 ± 1,5a	*F* = 13,587	<0.001
	6,2	5,1	6,3	4,6		
	(2,7-11,0)	(2,3-10,9)	(2,7-11,0)	(2,3-10,9)		
Lateral incisor region—first molar region (left)	21,2 ± 3,3b	17,9 ± 4,3b	21,3 ± 3,4b	18,3 ± 4,0a	*F* = 11,686	<0.001
	21,2	18,0	21,2	17,9		
	(15,2-28,0)	(8,3-26,7)	(15,2-28.0)	(11,7-28,0)		
Lateral incisor region—first molar region (right)	20,8 ± 3,3b	17,5 ± 4,1a	20,9 ± 3,3b	18,3 ± 3,9a	*F* = 10,998	<0.001
	20,3	17,8	20,3	18,1		
	(14,4-28,9)	(5,3-27,5)	(14,4-28,0)	(11,1-27,5)		
Lateral incisor region (left)—lateral incisor region (right)	19,0 ± 2,4b	15,4 ± 2,4a	19,0 ± 2,4b	15,7 ± 3,0a	*F* = 30,407	<0.001
	18,9	15,3	18,9	15,4		
	(14,0-26,1)	(10,3-21,8)	(14,0-26,1)	(8,9-22,7)		
Nasal floor—alveolar crest (right)	14,6 ± 3,5b	12,2 ± 3,6a	14,6 ± 3,5b	12,2 ± 2,9a	*F* = 8,031	<0.001
	14,5	12,2	14,4	12,5		
	(7,1-24,7)	(5,5-19,8)	(7,1-24,7)	(5,1-18,1)		
Nasal floor—alveolar crest (left)	15,0 ± 3,7b	12,5 ± 3,5a	15,0 ± 3,7b	12,0 ± 2,9a	*F* = 10,364	<0.001
	14,3	12,5	14,3	12,0		
	(6,7-25,4)	(5,4-21,2)	(6,7-25,4)	(5,3-18,0)		

Note: *F*: analysis of variance test statistics. Data are presented as mean value ± standard deviation/median (minimum-maximum) in millimeter. a-b: there is no difference between groups with the same letter (*p* < 0.05).

**Table 3:** Comparison of the nasal floor alveolar crest and lateral incisor region first molar region groups.

Experienced		Experienced CBCT	Inexperienced Panoramic	Inexperienced CBCT	Total	Test statistics	*p*
Panoramic							
Nasal floor—alveolar crest (right)						*χ* ^2^ = 12,382	0.006
<10	3 (6)a	13 (26)b	3 (6)a	10 (20)ab	29 (14,5)		
≥10	47 (94)	13 (26)b	47 (94)	40 (80)	171 (85,5)		
Nasal floor—alveolar crest (left)						*χ* ^2^ = 11,736	0.051
<10	3 (6)	12 (24)	3 (6)	11 (22)	29 (14,5)		
≥10	47 (94)	38 (76)	47 (94)	39 (78)	171 (85,5)		
Lateral incisor region—first molar region (left)						*χ* ^2^ = 23,570	<0.001
<15	0 (0)a	11 (22)b	0 (0)a	10 (20)b	21 (10,5)		
≥15	50 (100)	39 (78	50 (100)	40 (80)	179 (89,5)		
Lateral incisor region—first molar region (right)						*χ* ^2^ = 18,620	<0.001
<15	1 (2)a	12 (24)b	1 (2)a	9 (18)b	23 (11,5)		
≥15	49 (98)	38 (76)	49 (98)	41 (82)	177 (88,5)		

Note:. *χ*^2^: chi-square test statistic. a-b: there is no difference between groups with the same letter (*p* < 0.05).

The article "Comparison of the Efficacy of the Panoramic and Cone Beam Computed Tomography Imaging Methods in the Surgical Planning of the Maxillary All-On-4, M-4, and V-4" was published in 2022. Journal: Biomed Res Int.

**Table 4:** Distribution of the lateral incisor region first molar region (right) groups according to the nasal floor alveolar crest (right) condition.

Group	Lateral incisor region—first molar region (right)	Nasal floor—alveolar crest (right)		Total	*p*∗
		<10	≥10		
Experienced panoramic	<15	0 (0)	1 (2,1)	1 (2)	1.000
	≥15	3 (100)	46(97,9)	49 (98)	
Experienced CBCT	<15	3 (23,1)	9 (24,3)	12 (24)	1.000
	≥15	10 (76,9)	28(75,7)	38 (76)	
Inexperienced panoramic	<15	0 (0)	1 (2,1)	1 (2)	1.000
	≥15	3 (100)	46(97,9)	49 (98)	
Inexperienced CBCT	<15	2 (20)	7 (17,5)	9 (18)	1.000
	≥15	8 (80)	33(82,5)	41 (82)	

∗Fisher's exact test.

**Table 5:** Distribution of the lateral incisor region first molar region (left) groups according to the nasal floor alveolar crest (left) condition.

	Lateral incisor region—first molar region (left)	Nasal floor—alveolar crest (left)		Total	*p*
		<10	≥10		
Experienced panoramic	≥15	3 (100)	47 (100)	50 (100)	—
Experienced CBCT	<15	5 (41,7)	6 (15,8)	11 (22)	0.105
Experienced CBCT	≥15	7 (58,3)	32 (84,2)	39 (78)	
Inexperienced panoramic	≥15	3 (100)	47 (100)	50 (100)	—
Inexperienced panoramic	<15	1 (9,1)	9 (23,1)	10 (20)	0.424
	≥15	10 (90,9)	30 (76,9)	40 (80)	

∗Fisher's exact test.

## Data Availability

The data used to support the findings of this study are available from the corresponding author upon request.
